# XGBoost-Based E-Commerce Customer Loss Prediction

**DOI:** 10.1155/2022/1858300

**Published:** 2022-07-31

**Authors:** Lin Gan

**Affiliations:** School of Economics and Trade, Anhui Vocational College of Defense Technology, Lu'an 237011, China

## Abstract

In recent years, with the rapid development of mobile Internet, more and more industries have begun to adopt mobile Internet technology, provide diversified wireless services, and further expand user activity scenarios. The core of reducing customer loss is to identify potential customers. In order to solve the problem of how to accurately predict the loss of customers, this paper put forward an invented method to verify and compared the model with the customer data of an e-commerce enterprise in China. According to the research results, the improved XGBoost algorithm can effectively reduce the probability of class I errors and has higher accuracy, among which the accuracy has increased by 2.8%. The prediction effect of customer groups after segmentation was better than that before segmentation, in which the probability of the occurrence of class I errors in the prediction of core value customers decreases by 10.8% and the accuracy rate increases by 7.8%. Compared with other classification algorithms, the improved XGBoost algorithm had a significant improvement in AUC value accuracy rate and other indicators. This fully shows that the XGBoost algorithm can effectively predict the loss of e-commerce customers and then provide decision-making reference for the customer service strategy of e-commerce enterprises.

## 1. Introduction

At a time when computer technology is advancing by leaps and bounds, the amount of data generated will grow by about 40% a year. The massive data accumulated in this way contain rich content and contain a huge amount of information. On the other hand, relying on machine learning theory algorithms and data mining methods, it is mainly divided into subjective and objective aspects. Subjectivity is where your interests lie, what your abilities are, and how influential you are; objectively, what the media reports is what they are willing to report and what they are willing to spread, and the public selectively accepts what they are willing to receive. Popular, commercial, and recreational features should be noted, the discovery of information and the extraction of knowledge are more convenient and economical than before, and the information obtained is richer and more accurate. It costs very little to find new economic growth points or the best treatment for incurable diseases. This has not only changed the way of thinking and method of scientific research but also brought a new mode of social life to mankind. For an enterprise or website, the presence of members is very important. Compared with ordinary users, members are often more valuable in services such as subscription and payment. Due to the instability of customers and the volatility of the market, members may choose to continue to subscribe or give up membership for various reasons. The reasons are varied and often unpredictable. This is what any website or mobile application should focus on. Studies show that the cost of absorbing a new customer is nearly four times more than the cost of retaining an old customer. Maintaining a good relationship with their own customers can bring hidden wealth to enterprises. Moreover, with the extension of the enterprise and customer relationship maintenance time, bring more and more benefits. Therefore, any company or enterprise should put the maintenance of its customers, especially old customers, in an important position, maintain a good relationship with old customers, and develop new customers. If it is predicted that members will lose, it is necessary to take appropriate measures to retain members and reduce the loss of the company. In addition, as one of the most common research fields of data mining, recommendation system has a wide range of applications. We can recommend suitable applications and content to users according to their historical information. Bai Xueyang, for example, conducted research on personalized book recommendation. Chen Junran used collaborative filtering algorithm to recommend movie content. Data mining is a science of studying data and obtaining useful information from data. Different from simple statistical analysis of data, data mining focuses on extracting unknown and hidden information from known data. In recent years, with the diversification of data collection methods and the gradual improvement of data storage capacity, data mining has gradually set off a boom and become a subject that attracts more and more people's attention. On the other hand, the continuous upgrading of machine learning-related technologies also makes the overall optimization of data mining, and the experimental results are getting better and better. In terms of the combination with various fields, data mining technology also shows its more and more extensive application. Data mining can describe what happened in the past, what is happening now, and what is likely to happen in the future. Let us say you have data on 10 million customers. In view of long-term development, a preliminary prediction of customer retention should be made, considering which customers will retain and which customers will lose. Predictive models in data mining can solve such problems. The main work of predictive models can be divided into two steps, as shown in Figure 1. First, a model is constructed using a large number of data of known tags. Then, the constructed model is used to predict the data of unknown tags. After predicting the future situation, problems can be found in time and preparations can be made in advance. Business can be optimized, the best decision scheme can be set, and the problems can be avoided in advance.

## 2. Related Works

Mei and Li combined the theory of customer relationship management with the theory of customer value and took the e-commerce enterprise customers as the research object, analyzed the online shopping behavior of customers, evaluated the value of customers, subdivided customers, and further constructed a reasonable loss prediction model [1]. At present, XGBoost algorithm is seldom used to model customer loss prediction in e-commerce industry. Combining random forest with XGBoost algorithm, Yang improved XGBoost and applied it to customer loss prediction for the problem of two kinds of error loss, which provides some reference for the application and improvement direction of the algorithm in the future [2]. In the analysis of customer value, Gu et al. considered the social behaviors of customers in the process of online shopping and constructed a new value evaluation model RFMI based on RMF model, which enriched the customer value theory of e-commerce industry to a certain extent [3]. It also provides valuable reference for Lalwani et al.'s follow-up study on the correlation between customer social attributes and loss state [4]. Empirical data are obtained from an e-commerce enterprise in China. Through the analysis of customer behavior characteristics and value, Li and Li constructed a customer value model to identify the high-value customers of the enterprise and then predicted the loss of customers [5]. Such customer segmentation is beneficial for enterprises to carry out low-cost precision marketing, so as to increase their earnings. Naser and Al-Shamery based the loss prediction model that is built on integrated learning algorithm XGBoost, which automatically compresses data and fragments data when there is a large amount of data to improve the operation efficiency and occupy less memory, so it can play a greater role in the actual big data application scenarios [6]. According to the actual application scenarios of e-commerce, Jiang et al. considered the different loss of two types of errors in the classification model, and the integrated learning algorithm XGBoost is improved to improve the rationality of model application and accuracy of prediction [7]. The purpose of the study is mainly in the following two aspects. Zhang and Dong analyzed the customer value of e-commerce enterprises and built the customer value evaluation model based on the consideration of customer social behavior. The customer group segmentation of e-commerce enterprises is carried out, which is convenient for enterprises to carry out more accurate and scientific customer segmentation and loss prediction [8]. Based on the improved integrated learning algorithm XGBoost, Purnamasari constructed an e-commerce customer loss prediction model to predict customer loss of customer segments and the possibility of value customer loss, so as to improve the accuracy of the customer loss prediction model and prepare for the enterprise to further take customer retention measures [9]. Avanija et al. combined the theory of customer relationship management with the relevant theory of customer value, taking the customers of e-commerce enterprises as the research object, analyzing the online shopping behavior of customers, evaluating the value of customers, subdividing customers, and further constructing a reasonable loss prediction model [10].

## 3. Method

There are three major indexes in the traditional RFM model, respectively: R (time of last purchase), F (the frequency of consumption in the recent period), and M (the total amount spent in the last period of time). The model starts from the consumption behavior of individual customers and sets up key indicators to measure the historical value generated by customers and the possible future value. The index data are easy to obtain and calculate. However, in the application scenario of e-commerce, the value model also has some defects due to the simplicity of the index, which are mainly shown as follows. (1) It only considers the individual behavior of customers and lacks consideration of the mutual influence between customers. (2) Without considering the weight of indicators in the model, the weight of the three indicators is regarded as the same, but in the actual situation, this way of calculating customer value is unreasonable. Now, in order to adapt to the market environment, the modern e-commerce industry has gradually changed. More and more companies are finding that consumer autobiographical advertising and consumer word-of-mouth can lead to more traffic and revenue. In order to tap the benefits of customer relationships, many e-commerce companies integrate relationships into the online buying process and facilitate communication through shared discount groups, giveaways, and more to understand consumers' personalities. This personal communication between consumers creates a social network. We refer to this new e-commerce model based on social network interactions such as social e-commerce. In this environment, consumer demand and behavior are subtle, and their benefits to businesses may change accordingly. Consumers are not satisfied with the simple buying process, but there is a greater need for sharing and acceptance. Survey studies have shown that consumers benefit not only economically and functionally but also economically and emotionally [11]. From the perspective of consumption sociology, consumption is not only a process in which customers pursue the maximization of personal utility but also a process in which they reproduce social relations. With the development of marketing technology, the commodities and services of enterprises are gradually endowed with specific cultural connotations, and consumption has gradually become a way for people to express social identity and pursue a sense of belonging. From the perspective of e-commerce enterprises, in the social network environment, customers' positive social behaviors can also bring indirect benefits to enterprises. For example, the sharing behavior of customers in the process of shopping can bring more traffic to e-commerce enterprises. Customers' positive comment behavior can create more word-of-mouth effect for enterprises. In addition, as the sales model with high profit margin and low price is more likely to motivate customers' self-communication behavior, some discount sensitive customers will become the preference of social e-commerce. Therefore, low-cost and low-income consumers are not only important customers of enterprises, but also need to consider the impact of low-cost consumers on other consumers. If a customer can exert great influence on other customers, the loss of this customer will greatly lead to the loss of other customers. Out of respect for the customer to bring the influence of social behavior, this paper defines the customer value measured by the original M model as the customer's personal value and defines the customer's benefit value to the enterprise in social behavior as the customer's social network value, that is, the positive influence of a customer on other customers, and considers adding quantitative indicators to describe this value in the M model. High-value customers in social networks mean that they interact with more neighboring customers and can bring more traffic to the enterprise, while their loss may also lead to the loss of other customers. Considering the personal value and social network value of customers comprehensively, we integrate the social network influence of customers into the RFM model to construct a new customer value model. First, based on the two dimensions of customer value and social network value, we formulate customer value to measure the needs of social network e-commerce business. Personal value is mainly reflected in customers' purchase behavior, that is, customers' profits contributed to enterprises by generating transactions. The value of social network is reflected in the positive word-of-mouth effect brought by customers in their interactions with other customers, which mainly include sharing, invitation, group comments, etc. There are R, F, and M indicators in the RFM model. By paying attention to customers' recent purchase frequency and purchase amount, customers' personal value can be well measured [12]. However, the model lacks indicators to measure the value of customers' social networks. In this paper, the customer's social network value is defined as I (influence) index, which is integrated into the RFM model to form a new value evaluation model RFMI. Among them, R index, F index, and M index can be calculated based on the customer's consumption record. Index I refers to the value of social networking that consumers create in their behavior, and we measure it with various social networking models. Interactions between online users on social networks can generate a wealth of information. By analyzing this behavioral data, the impact of consumer behavior can be measured. In 2009, based on the analysis of log data, Goya Amit proposed a model to quantify the influence of users and behaviors, as shown in equations (1) and (2).

(1) $$\begin{array}{c} \inf\;l\left(u\right)=\frac{|\left\{a|\exists v,\Delta t:\text{prop}\left(a,v,u,\Delta t\right)\Lambda 0\leq \Delta t\leq r_{v,u}\right\}}{A_{u}}, \end{array}$$

(2) $$\begin{array}{c} \inf\;l\left(a\right)=\frac{|\left\{a|\exists v,\Delta t:\text{prop}\left(a,v,u,\Delta t\right)\Lambda 0\leq \Lambda t\leq r_{v,u}\right\}}{U\left(a\right)}, \end{array}$$

where *u* and *v* represent different customers, *a* represents actions, *∆t* represents the time interval between actions, and *t*_*vu*_ is a time constant. prop(*a*, *v*, *u*, Δ*t*) represents the propagation of actions between customers. *Au* two represents the number of actions generated by customer *u*, and *U*(*a*) represents the number of customers that generate actions [13]. Equation (1) describes the influence of user *u* as the ratio of the number of actions transmitted over a period of time to all actions produced by user *u*. Equation (2) describes the effect of behavior on the percentage of users who receive transmissions from each user over a period of time. Due to the limitation of information acquisition, this paper is only used to understand the sharing behavior of users. Regarding the concept of Goya Amit, we communicate the sharing behavior of customers through the products or activities shared by some users being clicked by other users. Due to the limitation of information acquisition, this document is only used to understand the sharing behavior of users. Using Goya Amit's idea for reference, we use the product or activity link shared by a customer to be clicked by other customers to express the sharing behavior that customer u has been spread. This paper quantifies the number of sharing rewards each customer has received from other different customers. Au II represents the number of sharing behaviors generated by customer u within a specific time. This can quantify the customer's social network value index I, as shown in formula (3). In this form, the number of gifts each customer shares with another consumer is counted. The second is about the number of behaviors generated by users in a specific time period, so that the user's social network value can be calculated, as shown in the following formula:

(3) $$\begin{array}{c} l_{u}=\frac{|\left\{a|\exists v,\Delta t:\text{prop}\left(a,u,\Delta t\right)\Lambda 0\leq \Delta t\leq r_{u}\right\}|}{Au}. \end{array}$$

At this point, we added I index to the original R, F, and M indexes of RFM to form a new value evaluation index system, as shown in Table 1.

The customer value identification model has three stages: index system construction, customer value calculation, and customer value classification, as shown in Figure 2. The first is the construction of the index system, that is, the value model of four indicators R, F, M, and I. Then, we determine the weight value of each major index through the expert scoring method. The consistency test of the judgment matrix is carried out. The second is the calculation of customer value, which uses the method of multiplication and addition to calculate the value of the relevant customer data that has been collected and processed, so as to get the value *v* of each customer. Finally, the customer value classification, that is, according to the calculation results of the second step and the distribution of customers, determine the threshold, and divide the customer categories according to the threshold. Different thresholds represent customers with different values [14].

In the RFMI model, the four indicators have different impacts on customer value, so the impact of different indicators on customers should be distinguished as far as possible in the setting of index weight. This paper uses analytic hierarchy process to solve the index weight problem in the RFMI model. Analytic hierarchy process (AHP) is a powerful and flexible decision-making tool for ensemble construction measurement and analysis. It is suitable for complex problems that need to consider both qualitative and quantitative aspects and has been widely used in various problem scenarios. Firstly, according to the final goal, the decision criteria are defined and the complete hierarchical structure is constructed, that is, the organization from the self-standard layer to the middle layer and then to the bottom layer is established according to certain standards. A simple pairwise comparison is then used to determine the rating and weight, and the rating importance is converted into a score through the scale. Finally, the problem is summed up as the determination of the relative importance weight of the lowest layer relative to the target layer. Establish a single-level model structure for the case study in this paper, as shown in Figure 3.

The maximum characteristic root *λ*max and its characteristic vector *W* of the judgment matrix are calculated, where *W* is the ordering weight of importance. To further test the consistency of the matrix, see formula (4) for defining the consistency index:

(4) $$\begin{array}{c} C1=\frac{\lambda \max-n}{n-1}. \end{array}$$

In order to measure the size of *C*1, *λ*max is the largest characteristic root, and *n* is the matrix reference index. We also introduce a random consistency index RIoRI, which is related to the discriminant matrix. In general, the greater the order of the matrix, the greater the probability of consistency deviation. The corresponding standard values are shown in Table 2.


(5) $$\begin{array}{c} \text{CR}=\frac{\text{CI}}{\text{RI}}. \end{array}$$

The consistency of the matrix can be measured by formula (5). If CR < 0.1, the matrix is considered to pass the consistency test; otherwise, the coefficients need to be readjusted until the matrix passes the consistency test. Customer value consists of personal value and social network value. In a certain period of time, the characteristics of customers' personal consumption, including consumption frequency and time, can be calculated from customers' consumption record data [15]. Social network value refers to the value brought by the social behavior generated by customers. This paper studies the sharing behavior in social behavior, and quantifies the customer's social network value with the customer's sharing data, which can be calculated by formula (3). Starting from the two dimensions of personal value and social network value, this paper divides customers into four categories, as shown in Figure 4.

*The First Quadrant*. Core value customers are those with high personal value and high social network value. Such customers have frequent transactions with the enterprise, large transaction volume, and frequent social behavior, which can bring more additional income for the enterprise. Maintaining the relationship with such customers can bring stable income to the enterprise and ensure its sustainable development. Customer relationships exist in every aspect of a business, but it is most prevalent in the customer service department. Customer service teams, customer support, customer success, and product development play an important role in building healthy customer relationships.

*The Second Quadrant*. Important value customers are those with high personal value but low social network value. For this kind of customers, we should strengthen customer relationship management to prevent their loss. Let us start with social networks first, and let us review some of the functions and driving forces provided by social networks behind the rise of social shopping. From a global perspective, we have some inspirations from the data provided by different market research institutions. Passing the 1.2 billion mark at the end of the year, the percentage of social network users in the Asia-Pacific region will be higher, and the social activity will be stronger. In the Asia-Pacific region, the number of social network users in China, a huge market, has risen to more than twice that of the United States this year. These customers are the traditional high-value customers of e-commerce enterprises and are often loyal customers of enterprises. They may not adapt to the shopping mode in the social network environment and thus have low social network value. On the other hand, social guiding operations can be added to guide the positive social behaviors of such customers and change their consumption habits, thus increasing the social network value of such customers.

*Third Quadrant*. General value customers are those with low personal value and low social network value. These customers are ordinary customers of enterprises with low purchase frequency and small transaction volume, and their latest transaction time is far from each other and they do not have high social network value. Therefore, their purchase behavior is mostly accidental. It is not recommended to invest too much resources in customer relationship maintenance for such customers [16].

*The W Quadrant*. Important development customers, namely, those with low personal value and high social network value, have low transaction frequency and small transaction volume but are willing to share and pay more attention to preferential promotion activities. Although such customers bring low direct profits to the enterprise, they can accumulate sales and online reputation for the enterprise, improve its popularity, and bring more new customers to the enterprise. This kind of customer has great marketing value for enterprises. Customer relationship management mainly includes three aspects, one is customer value, the other is customer relationship value, and the third is information technology. The goal of customer relationship management is to maximize customer value. For any company, the purpose of customer relationship management is to maximize customer value, improve customer satisfaction, allow customers to recognize the products or services provided by the company, enhance the customer's recognition and loyalty to the enterprise, and develop long-term customer relationship with each other. For such customers, enterprises can enhance customer contact while excavating their marketing value and take marketing measures to improve customer stickiness so as to convert them into higher-value customers. In order to classify these four types of customers more intuitively, we define customer value *U*. Customer value *V* is the sum of personal value and social network value, and its calculation formula is shown in equation (6). When the index value obtained in the data processing stage (after standardized processing) and the weight *W*_*i*_ of each index determined by analytic hierarchy process are substituted into the value calculation formula, the value of each customer can be calculated. Then, according to the actual situation of the enterprise and the proportion of customers, it determines the proportion of high-value customers *P* and then determines the value of the *n∗P* customer (n is the total number of customers), which is denoted as *V*_*n∗P*_. The customer whose value is higher than *V*_*n∗P*_ is regarded as the core value customer of the enterprise. Then, remove the core value customers and identify the important value customers in proportion, and so on, until the customer classification work is complete [17]:

(6) $$\begin{array}{c} V=W_{1}*\left(\frac{1}{R}\right)=W_{2}*F+W_{3}*M=W_{4}*I. \end{array}$$

The smaller the *R* value is, the more recent the customer's last purchase is and the higher its value is, so we use its reciprocal in value calculation formula (6) for calculation. The customer value identification model constructed above is applied to the e-commerce customer classification scenario, and the rationality of the model is verified by the customer segmentation results. The application process of the model and the customer segmentation results will be specified below.

## 4. Experiments and Analysis

Python is currently the most widely used programming language in data science, and it has many advantages. First of all, Python has a simple syntax that makes it very novice friendly, and it works with other languages, such as Java and C. Moreover, there are rich libraries for data analysis and distributed computing, and a steady stream of scholars have packaged algorithms into libraries and published them for everyone to use. Up to now, these algorithms have reached more than one hundred thousand, greatly convenient for data analysis work, so that the original obscure algorithm can be realized through black box operation, such as numpy, pandas, scikit-learn, and so on. Pandas and scikit-learn have great advantages in data analysis. Pandas can handle the early data processing, and scikit-learn not only packages rich algorithms, such as logistic regression, decision tree, support vector machine, and random forest (which we use most often), but also provides many methods for feature selection. The two methods used above are implemented using this powerful library [18, 19]. In this experiment, the user behavior data of 1 to 6 months is used as the total training set, and the length of the training set selected for each training is increased (the data of June is used as the training set for the first time, the data of May and June are used as the training set for the second time, and so on, and the size of the training set is gradually increased from 1 month to 6 months), so as to predict the loss of users in the seventh month. This experiment was repeated for 3 times, and the user loss in July, September, and September was predicted with the sliding of the mobile window for 3 times. The average prediction results obtained in the end are shown in Figure 5.

As shown in Figure 5, the *x*-axis represents the span of months of training data, and the *y*-axis represents the performance indicators of the customer loss prediction model, including precision, recall, AUC, and *F*1-score. In general, it can be said that large samples of training data can improve the effect of the model. In terms of *F*1-score, a larger sample of training data achieved an improvement of about 17, and this proves the importance of data volume in customer loss research. This result also suggests that data stored for at least four or five months are needed to train attrition forecasting models to achieve better attrition forecasting results [20]. In the following experiment, the user data with a span of four months will also be selected as the training set. However, it is more noteworthy that the precision, recall and *F*1-score curves show that the returns of the prediction model decrease with the increase of the time span of the training set. This is normal for the relationship between data volume and predictive performance, especially for linear models such as logistic regression. There are two possible reasons for this. On the one hand, the model may be too simple to capture the characteristics of the larger dataset. On the other hand, the data accumulated in the past few months or the earlier data used to train the model may not be useful for predicting the potential loss of users in the latest month [21]. For example, the customer loss behavior in the first month may not be correlated with the customer loss behavior in the seventh month, that is to say, the reasons for customer loss in the first month are different from those in the seventh month. This phenomenon also follows the first-order Markov property: the current state depends only on the closest previous state. In the model of customer loss prediction, increasing the sample size of the training set can improve the effect of the model. From another perspective, for the training set that determines the sample size of the training set, increasing the number of features of each sample is another method to increase the data of the training set. The author believes that if there are more features that provide a small but non-zero amount of additional information about the predicted target, the effectiveness of the prediction model can benefit from a wide variety of features [22]. In terms of user basic features, 32 features (information based on BBS system functions) F1 are obtained through dimension reduction of trestle automatic encoder. Other features added one by one including feature F2 from CS module to express user mobile communication service related information, feature F3 from PS module to express user mobile data service information, F4 to express the function of user call graph, feature F5 to express user short message graph, feature F6 to spread information based on user relationship, natural language feature F7 for customer service and complaint, and the topic word feature F8 for search query. A detailed description of these characteristics can be found in Section 4.1. In the dataset in Table 1, the experiment was repeated for 5 times to predict the loss from the 5th to 9th month. The user data marked in the first four months of the prediction target was used as the training set and the potential loss in the next month was predicted. The average result of the evaluation index of the prediction effect is shown in Table 3.

The above experimental data summarize the impact of each new feature on customer loss prediction model. It can be seen that the features (*F*2 and *F*3) composed of CS module information reflecting users and PS module information reflecting users have significantly improved AUC. This result suggests that these two features are very effective in predicting customer loss because customer loss behavior is closely related to voice and data services. Customer-centric network optimization solutions can be used in experiments to improve the KPI/KQI experience of potential loss users. It can also be seen that PS module features are more effective than CS module features in customer loss prediction because customers are using more and more mobile data services in China, and voice services are becoming less important than before. Surprisingly, the features from customer service and user complaint related information (F7) and the feature based on SMS relationship graph (F4) contribute the least to the effect of customer churn prediction model because almost all customers use wechat, Dingding, and other applications and rarely use SMS services. In contrast, the function of user call graph (*F*4) and user loss propagation graph (*F*6) can improve prediction performance more than the function based on message graph. The importance of the user churn communication graph shows that customers with relevance tend to churn with similar possibilities. For example, college students have strong edge power in the co-occurrence chart and often lose at the same time. Or, represented by family users and company users, when one of them stops using a certain business product, other related users will also lose behavior. The thematic features of customer service and complaint text messages (*F*7) from users did not improve significantly for the prediction model, suggesting that complaints from users were not a major early signal. Although the majority of lost users have a bad experience, they still do not actively seek customer service or complain before losing. In contrast, the subject function of the search query (*F*8) is more informative. Potential loss can visit other carriers' portals, search other carriers' hotlines, search for new phones, and so on. In addition, graph-based features also play an important role in distinguishing attrition users from non-attrition users [23]. In fact, attrition users influence non-attrition users through phone calls, text messages, and real relationships, especially in terms of user relationships. Other display features include some high-order features that are difficult to define. Although the phenomena corresponding to reality cannot be seen through the nature of the data, they also play an important role in experimental results. The above results suggest that OSS system information can improve the accuracy of loss prediction and it is valuable to integrate BSS and OSS data into prediction modeling [24, 25], as shown in Figure 6.

Data imbalance is an obvious problem for customer loss forecasting model. The experimental purpose of this section is to explore the influence of different sampling methods on customer loss prediction model [26, 27]. In this experiment, there are four methods to deal with data imbalance: (1) imbalance; (2) Random upsampling; (3) SMOTE; and (4) SMOTE Tomek-link. The first approach trains the model directly with unbalanced dataset instances. The second method randomly replicates instances of a small number of samples (lost customers) until the two samples have the same number. The third method is different from random upsampling in that it creates similar samples in a few classes instead of duplicating repeated samples, so as to achieve the goal that the number of samples in a few classes is close to the number of samples in most classes. In the fourth method, similar samples are created in a few classes first, and then boundary samples close to the few classes are deleted from the majority of classes (non-attrition users). In the samples obtained by four different sampling methods, the trestle self encoder is used to reduce the feature dimension to 32 features, add other features of F2 to F8, use the user data marked in the first four months of the prediction target as the training set, and predict the potential lost users in the next month. In the XG boost and random forest model, the experiment is repeated five times to predict the lost users from May to September. The random forest uses the Gini index decision tree as the base learner, and the maximum depth is set to 20 to avoid overfitting.  Table 4 shows the average results of the five tests [28]. The result pairs of the oversampling method under the XGBoost model are shown in Table 4.

The result pairs of the oversampling method under the random forest model are shown in Table 5.

By comparing the above results, it can be seen that the model effect accuracy of unsampled unbalanced data as a training set is higher than the dataset effect of other upsampling methods. On the contrary, the model recall rate obtained by the training of other datasets is higher than 80%, among which the model trained by the random upsampling method is slightly better than the results of the training of the other two datasets. It can be seen that although the random upsampling method has a simple idea, it has a high degree of data fit for customer loss. Therefore, it is recommended to use the random upsampling method to deal with unbalanced datasets in the research on customer loss prediction.

## 5. Conclusion

Customer loss management is one of the important links in enterprise customer relationship management. Facing the problem of customer loss, the primary task of e-commerce enterprises is to identify the potential customer loss and then take corresponding measures in advance to reduce the loss as far as possible in order to maximize their own interests. Existing research shows that customer segmentation can improve the accuracy of churn prediction of high-value customers. In addition, during the research process, this paper finds that there are few relevant studies on customer value analysis considering social behavior, and there are many dimensions and large quantities of customer data in e-commerce enterprises, which are the main challenges for enterprises to predict customer churn at present. In view of the deficiencies of existing research, this paper provides a user value proposition and distribution model to determine the value of consumer consultation and designs a stochastic prediction model combining random forest and XGBoost learning algorithm to solve the e-commerce gambling problem. The research conclusions of this paper are as follows. In view of the development characteristics of e-commerce industry, this paper deeply analyzes the value of e-commerce customers and constructs a value evaluation model RMFI considering customer social behavior to carry out customer segmentation work, help enterprises identify value customers, and create prerequisite conditions for differentiated precision marketing. The results show that although the number of core value customers is small, they contribute to the majority of profits of enterprises, while the high proportion of general customers and low proportion of consumption can create little profit for enterprises. In order to achieve reasonable allocation of resources, enterprises should give priority to the management and operation of core value customers.

The improved algorithm has better performance. In this paper, according to the characteristics of e-commerce customer loss problem, random forest and XGBoost algorithm are combined to build a loss prediction model, and the loss function of XGBoost algorithm is improved. It is found that the random forest feature selection method can effectively solve the problem of too many data dimensions caused by too many factors affecting customer churn, and the improved integrated learning algorithm xgboost can not only be well applied to big data scenarios without efficiency loss but also reduce the probability of misjudgment of lost customers, that is, reduce the probability of a class of errors and optimize the overall prediction effect. The combination of user segmentation and customer prediction can improve the predictive ability of the XGBoost algorithm. This paper divides consumer groups according to consumption value and then uses a fall prediction model to estimate the loss of consumer groups before and after the segmentation. The research results showed that after customer segmentation, all indicators of the prediction result were significantly improved, among which the prediction accuracy of core value customers was increased by 7.8% and AUC value was increased by 6.3%; this also verifies the effectiveness and value of XGboost algorithm in e-commerce customer churn prediction.

## Figures and Tables

**Figure 1:** XGBoost-based e-commerce customer loss prediction.

**Figure 2:** Customer value identification model framework.

**Figure 3:** Single hierarchy analysis chart of customer value.

**Figure 4:** Customer classification dimension.

**Figure 5:** The influence of training set size on prediction results.

**Figure 6:** The influence of feature number on prediction results.

**Table 1:** Customer and value evaluation system.

Target	Dimensionality	Index	Definition of indicator
Customer value evaluation	Personal value	R (recency)	Most recent purchase time
		F (frequency)	Purchase frequency
	Social network value	M (monetary)	Total consumption
		I (influence)	Influence on other customers

**Table 2:** RI reference standard value corresponding to matrix sequence.

The matrix order	1	2	3	4	5	6	7

RI	0	0	0.58	0.9	1.12	1.24	1.32

**Table 3:** The influence of feature number on experimental results.

Features	AUC (%)	Recall (%)	Precision (%)	*F*1-score
*F*1	89.47	71.25	28.13	40.34
*F*1&*F*2	93.50	80.81	37.51	51.24
*F*1&*F*3	93.84	81.07	38.71	52.40
*F*1&*F*4	91.45	76.20	34.99	47.96
*F*1&*F*5	89.86	72.10	28.54	40.89
*F*1&*F*6	92.47	78.80	35.78	49.21
*F*1&*F*7	90.66	72.82	29.77	42.26
*F*1&*F*8	91.02	76.02	34.18	47.16

**Table 4:** Results of oversampling method under the XGBoost model.

Dataset	AUC/%	Recall rate/%	Precision/%	*F*1-score
Random oversampling	97.78	90.59	31.51	46.76
SMOTE	97.46	89.11	30.68	45.64
SMOTE&Tomek-link	97.79	91.03	31.66	46.98
DATAIMBALANCED	85.38	73.99	43.00	54.39

**Table 5:** Results of oversampling method under random forest model.

Dataset	AUC/%	Recall rate/%	Precision/%	*F*1-score
Random oversampling	97.62	88.94	33.28	48.44
SMOTE	97.3	88.56	34.95	50.12
SMOTE&Tomek-link	97.41	88.98	34.61	49.84
DATAIMBALANCED	88.38	74.12	35.12	47.66

## Data Availability

The data used to support the findings of this study are available from the corresponding author upon request.
